# Increased survival and cell cycle progression pathways are required for EWS/FLI1-induced malignant transformation

This article has been retracted.

**DOI:** 10.1038/cddis.2016.268

**Published:** 2016-10-13

**Authors:** Tahereh Javaheri, Zahra Kazemi, Jan Pencik, Ha TT Pham, Maximilian Kauer, Rahil Noorizadeh, Barbara Sax, Harini Nivarthi, Michaela Schlederer, Barbara Maurer, Maximillian Hofbauer, Dave NT Aryee, Marc Wiedner, Eleni M Tomazou, Malcolm Logan, Christine Hartmann, Jan P Tuckermann, Lukas Kenner, Mario Mikula, Helmut Dolznig, Aykut Üren, Günther H Richter, Florian Grebien, Heinrich Kovar, Richard Moriggl

**Affiliations:** 1 Ludwig Boltzmann Institute for Cancer Research, Vienna, Austria; 2 Institute of Animal Breeding and Genetics, University of Veterinary Medicine, Vienna, Austria; 3 Medical University of Vienna, Vienna, Austria; 4 Center of Physiology and Pharmacology, Vienna, Austria; 5 Clinical Institute of Pathology, Vienna, Austria; 6 Children's Cancer Research Institute, St. Anna Kinderkrebsforschung, Vienna, Austria; 7 CeMM Research Center for Molecular Medicine of the Austrian Academy of Sciences, Vienna, Austria; 8 Department of Pediatrics, Medical University of Vienna, Vienna, Austria; 9 Randall Division of Cell and Molecular Biophysics, King's College London, London, UK; 10 Department of Bone and Skeletal Research, Institute of Experimental Musculoskeletal Medicine, University Hospital Münster, Münster, Germany; 11 Institute of General Zoology and Endocrinology, University of Ulm, Ulm, Germany; 12 University of Veterinary Medicine, Vienna, Austria; 13 Institute of Medical Genetics, Vienna, Austria; 14 Georgetown University Medical Center, Lombardi Comprehensive Cancer Center, Washington, USA; 15 Children's Cancer Research Centre and Department of Pediatrics, Klinikum rechts der Isar, Technische Universität München, Munich, Germany

## Abstract

Ewing sarcoma (ES) is the second most frequent childhood bone cancer driven by the EWS/FLI1 (EF) fusion protein. Genetically defined ES models are needed to understand how EF expression changes bone precursor cell differentiation, how ES arises and through which mechanisms of inhibition it can be targeted. We used mesenchymal Prx1-directed conditional EF expression in mice to study bone development and to establish a reliable sarcoma model. EF expression arrested early chondrocyte and osteoblast differentiation due to changed signaling pathways such as hedgehog, WNT or growth factor signaling. Mesenchymal stem cells (MSCs) expressing EF showed high self-renewal capacity and maintained an undifferentiated state despite high apoptosis. Blocking apoptosis through enforced BCL2 family member expression in MSCs promoted efficient and rapid sarcoma formation when transplanted to immunocompromised mice. Mechanistically, high BCL2 family member and CDK4, but low P53 and INK4A protein expression synergized in Ewing-like sarcoma development. Functionally, knockdown of *Mcl1* or *Cdk4* or their combined pharmacologic inhibition resulted in growth arrest and apoptosis in both established human ES cell lines and EF-transformed mouse MSCs. Combinatorial targeting of survival and cell cycle progression pathways could counteract this aggressive childhood cancer.

Ewing sarcoma (ES) is a highly metastastatic bone and soft tissue tumor with poor survival rates. The malignancy is caused by fusion of chromosome 11 and 22 creating the EWS/FLI1 (EF) transcription factor. EF expression is important for ES maintenance and compounds targeting EF protein are being developed for clinical applications.^1, 2, 3, 4^ To study EF expression with a mouse model that faithfully resembles ES development remains difficult owing to high toxicity induced by EF. It is controversial if EF expression alone is sufficient to promote ES or if it requires cooperating mutations. Despite EF-induced toxicity, murine or human mesenchymal stem cells (MSCs) tolerate expression, but only murine EF-transduced MSC displayed sarcoma formation upon transplantation in immunocompromised mice.^5, 6, 7, 8^ One lentiviral overexpression approach identified ERG-expressing embryonic superficial zone cells from murine cartilage as sarcoma stem cell origin.^7^ Tumor formation was influenced by positional effects of lentiviral vector integration into cancer-associated gene loci, but a unified hotspot integration was not reported.^7^ Zebra fish-mediated EF or endogenous EWSR1- or Rosa26-promoter-driven EF expression in mice promoted high apoptosis induction preventing ES.^9, 10, 11^ Although high EF expression caused embryonic lethality, moderate EF expression in two transgenic founder lines was associated with mild, but consistent limb shortening with normal life span without ES appearance. Compound cross with p53-deficient mice (*Prx1Cre*-mediated p53 deletion) synergized in osteosarcoma formation.^12, 13^ Furthermore, data from six independent laboratories presented 16 different Cre-mediated transgenic approaches to generate an Ewing Sarcoma mouse, which failed owing to high apoptosis and toxicity upon EF expression in multiple cell types.^14^

We aimed to better model the cellular origin of ES and we used *Prx1Cre* (EF^Prx1^) mice, which facilitated EF expression to early mesenchymal progenitors. EF expression caused a bone differentiation arrest owing to changed developmental signaling. As a result, severe malformations of the skull, facial bones, sternum and limbs and early perinatal death occurred. EF-immortalized MSC-like cells isolated from EF^Prx1^ limbs displayed high levels of apoptosis but failed to form ES. However, when cells were transduced by retrovirus to express BCL2 family members, they formed efficiently sarcomas in NSG mice. Sarcomagenesis was accompanied by upregulation of the CDK4/cyclin D1/pRB axis, and reduced INK4A and P53 expression accelerating cell cycle and survival. Depletion of *Mcl1* or *Cdk4* in a panel of EF-dependent cell lines led to inhibition of cell proliferation and enhanced apoptosis. Combined blockade of MCL1 and CDK4 with pharmacologic inhibitors caused cell cycle arrest and apoptosis in EF-transformed cells.

## Results

### Skeletal defects in EF^Prx1^ mice are due to blocked bone differentiation

We limited EF expression to early mesenchymal progenitors using Prx1Cre (EF^Prx1^) to better model the cellular origin of ES. To regulate EF expression in target tissues we used an EF expression cassette flanked by a floxed STOP cassette knocked into the Rosa26 locus.^10^ Compound mice with conditional mesenchymal *Prx1Cre* recombinase expression (Figure 1a) were generated. *Prx1Cre*-mediated recombination was reported from E9.5 onwards in bone-forming cells.^13^ Prx1 promoter-driven EF expression was shown to be tolerated, which resulted in shortened limbs upon transgenic expression, but detailed bone development was not analyzed.^12^ Here, we aimed to express EF during early development, as cases of congenital ES in newborns exist.^15, 16^ EF expression caused developmental abnormalities such as endochondral bone formation arrest, starting at E10.5 up to postnatal day P1 (Figure 1). EF-expressing embryos or newborns displayed gross malformations in limb development that became apparent at E12.5. The phenotype was more prominent from anterior-to posterior and at later developmental stages (Figure 1b; Supplementary Figure 1a–c). Malformations in rib cage architecture and in the craniofacial area most likely led to death of EF^Prx1^ newborn mice within the first 24 h postnatal owing to breathing and nutrition problems. Spine development remained normal (Supplementary Figure 1d). Alcian Blue/Alizarin Red staining, which stains cartilage in blue and bone elements in red, and skeletal analysis displayed severe reduction in calcified deposition (red elements) of long bones in EF^Prx1^ *versus* wild-type (wt) limb bones at E16.5. Furthermore, we observed a distorted sternum with deranged ossification center, causing an open, malformed rib cage. Calvaria bones lacked significant calcification, leading to skull malformations (Figure 1b). Mutant mice were born at normal Mendelian ratios (*n*=174 EF^Prx1^ *versus n*=161 wt controls were analyzed; Figure 1c). Detailed histological analysis of E13.5 and E18.5 embryos revealed two different phenotypes in limbs. All mutant embryos analyzed showed condensed cartilaginous elements instead of long bone formation. Although ~90% of mutants displayed polydactyly, only ~10% EF embryos lacked digits or long bone elements (Figure 1d; Supplementary Figure 1e). Van Kossa/Alcian Blue staining of E13.5 and E18.5 embryos revealed blocked mesenchymal differentiation in EF^Prx1^ mice at the pre-hypertrophic chondrocyte stage. In line, all mutant embryos showed absence of hypertrophic and mature chondrocytes or osteoblasts as confirmed by RNA *in situ* hybridization for bone lineage markers. Interestingly, although early markers of the chondrocyte lineage (*Sox9*, *Collagen 2a1*, *Col2a1*) were expressed in EF^Prx1^ limbs, markers of hypertrophic chondrocytes and osteoblast differentiation (*Indian hedgehog*, *Ihh*; *Collagen10*, *Col10a1*; *Runt-related transcription factor 2*, *Runx2* and *Osterix*, *Osx*) were largely absent in long bone areas, but weakly expressed in polydactyly digits. In rare cases, EF embryos lacked both digits and limbs, best visible by condensed *Collagen 2a1-*expressing cartilage elements at late development (Figure 1d; Supplementary Figure 3a). Similarly, osteoblast markers *Col1a1* and *Osc* were absent in limbs isolated from EF^Prx1^ embryos, but expressed in wt limbs (not shown). Immunoblotting analysis confirmed significant EF expression in limb elements (Figure 1e). Efficient deletion of the STOP cassette and expression of EF was confirmed by genomic or real-time PCR (Supplementary Figure 2).

### Impairment of bone development pathways in EF^Prx1^ limbs

EF^+^ embryos at different embryonic stages (E14.5, E16.5 and P1) showed a severe reduction of mature chondrocytes in mutant limbs, as measured by dimethylmethylene blue staining, which reflects sulphated glycosaminglycane content (Figure 2a; Supplementary Figure 3b). The WNT/*β*-catenin pathway has a pivotal role in chondrocyte and osteoblast differentiation in cooperation with BMP/SMAD and TGF-*β* signaling.^17, 18, 19, 20, 21, 22^ We analyzed by immunostaining key marker proteins (*β*-CATENIN, SMAD1/5, pSMAD4, SMAD7, DLX5, SOX9, RUNX2 and OSTERIX) along bone differentiation markers. Automated quantification of immunostaining served as reliable source to quantify levels.^23^ RUNX2, OSTERIX, DLX5, pSMAD4, SMAD1/5, SMAD7 and *β*-CATENIN were found diminished at all embryonic stages in EF^Prx1^ transgenic limbs (Figures 2a and b; Supplementary Figure 4), whereas SMAD7 expression at birth was comparable with wt expression levels. SOX9 expression for pre-hypertrophic chondrocyte differentiation, controlling secretion of extracellular matrix molecules like collagen and proteoglycans^24^ was normal during early development. DLX5 as a TGF-*β*-induced protein was downregulated in mutant limbs compared with controls (Figures 2a and b; Supplementary Figure 4).

### High level of apoptosis in limb elements of EF-expressing newborns

Next, we investigated EF expression and highest expression was seen at E14.5 and E16.5, whereas its expression diminished at P1 (Figures 3a–c; Supplementary Figure 5). The proliferation rate of EF-mutant chondrocytes was not significantly changed, as measured by Ki67 staining. However, TUNEL staining showed marked rates of apoptosis at P1 in mutant but not wt limbs (Figures 3a–c; Supplementary Figure 5). Of note, nuclear P21 (CDKN1A), a known senescence marker often lost or mutated in human cancer^25^ was induced at E14.5, but suppressed from E16.5 on in EF-mutant limbs. Moreover, cyclin D1 expression was slightly decreased throughout development of EF^Prx1^ transgenic limbs, whereas its expression was diminished at birth (Figures 3a–c; Supplementary Figure 5).

### EF-expressing MSCs are immortal and fail to differentiate

To study primary cells of malformed bone elements, 12 different primary EF^Prx1^MSC-like cell cultures (MSCL) from individual P1 EF^Prx1^ (EF^Prx1^MSCL) or six wt limbs (wtMSCL) as controls were propagated (Figure 4a; Supplementary Figure 6a–c). We applied specific differentiation protocols for osteoblasts, chondrocytes or adipocytes. WtMSCL cells displayed prominent differentiation into all three lineages, but EF^Prx1^MSCL reproducibly failed to differentiate (Figure 4a). Transgene expression of EF at the RNA- and protein level in EF^Prx1^MSCL cultures was verified and cells expressed CD90 (Thy-1.1) as a MSC marker (Figure 4b). Furthermore, mRNA expression for TGF-*β* receptor chains (*TgfbrI* or *TgfbrII*) and bone differentiation markers *Ostx, Sox9*, *Runx2, Osc* and *Dlx5* as the osteoblast differentiation master regulator was decreased in EF^Prx1^MSCL, whereas expression of hedgehog signaling components *Gli1*, *Ihh* and *Smo* was elevated. *P53* and *c-myc* were comparable to controls (Figure 4c; Supplementary Figure 6d; P53 protein level was also similar, not shown). WtMSCL displayed growth arrest after ~6–8 passages with senescence-like features such as PML^+^ immunostaining (not shown). In contrast, mutant EF^+^MSCL were continuously passaged (>50 passages). We did not observe senescence in EF^Prx1^MSCL and cells remained diploid even at passage 55. Cell cycle analysis of multiple different primary EF^Prx1^MSCL lines at early and late passage numbers (passage 8 and 55) displayed a large fraction (>40%) of cells at sub-G1 at early passage, but high rate of apoptosis was lost at late passage. Apoptosis loss was associated with a higher number of cells that remained in G2/M phase compared with wtMSCL (Figure 4d). High level of apoptosis in EF^Prx1^MSCL cells correlated with high *Caspase-3* mRNA levels (Figure 4d) paralleled by >80% TUNEL^+^ cells in limb elements at P1 of EF^Prx1^ newborns.

### Enforced BCL2 family member expression promotes sarcoma formation

We suspected that BCL2 family member expression in ES could be high. Indeed, all three family members, MCL1, BCL2 and BCL-x_*L*_ in ES cell lines SK-N-MC, TC71, TC252 and A673 were prominently expressed by Western blot analysis. Levels of protein expression were comparable to colorectal cancer cell lines HT29, HCT116, SW620 and LS174T, which are known to rely on high BCL2 family member expression to maintain viability.^26^ We also checked CDK4 expression in ES cell lines as a proliferation marker, which was upregulated compared with control cells (human prostate epithelial RWPE-1 cells; Figure 5a). EF^Prx1^MSCL were unable to promote sarcomagenesis when 4 × 10^6^ cells embedded in matrigel were s.c. injected into NOD.Cg-*PrkdcscidIl2rgtm1Wjl/SzJ* (NSG) recipients. We kept EF^Prx1^MSCL continuously in culture for more than 1 year and despite high passage number (>55 passage), we failed to detect tumourigenesis in NSG mice (Figure 5b). We conclude that primary EF^Prx1^MSCL cell lines are immortal and differentiation-resistant, but incapable to initiate sarcomas. BCL2 family members are proto-oncogenes and they promote survival and facilitate proliferation of cancer cells.^27^ Therefore, we examined if exogenous provision with *Bcl2, Bcl-x*_*L*_ or *Mcl1* could promote sarcomagenesis. We transduced *Bcl2, Bcl-x*_*L*_ and *Mcl1* by retroviral means (Bcl2-IRES-eGFP, Bcl-x_*L*_-IRES-eGFP, Mcl1-IRES-eGFP or GFP-vector control) in primary EF^Prx1^MSCL or wtMSCL lines to test their transforming capability. All transduced EF^Prx1^MSCL cell lines with BCL2 family members gave rise to prominent sarcoma formation within 3–4 weeks and with 100% penetrance when 4 × 10^6^ Bcl2-, Bcl-x_*L*_- or Mcl1-transduced EF^Prx1^MSCL cells were injected. WtMSCL with or without BCL2 family member transduction or GFP-vector transduced EF^Prx1^MSCL cells did not form any tumor. All transplanted cells were embedded in matrigel to enhance engrafting and NSG mice of control groups were followed up to 6 months. Consistently, high tumor burden and growth rate was found with any of the BCL2-transduced EF^Prx1^MSCL (Figure 5b; Supplementary Figure 7a and b). Remarkably, EF^Prx1^MSCL+Bcl2 cells were more invasive with higher tumor weight, whereas EF^Prx1^MSCL+Mcl1 cells expanded along the skin and muscle areas (Supplementary Figure 7a). Histo-pathology analysis of sarcoma sections confirmed a Ewing-like sarcoma morphology (Figure 5c; Supplementary Figure 7c). All sarcomas showed uniform small blue round cells with prominent nucleoli surrounded by small cytoplasm. Next we tested sarcoma cells for two established ES markers: periodic acid schiff (PAS) and neuronal-specific enolase (NSE) immunostaining confirmed ES-like staining pattern (Figure 5c; Supplementary Figure 7c).

### MCL1 transduction resembles a close human ES gene expression profile

To determine the similarity in gene expression of the transplant model with human ES we performed RNA-seq analysis. Data were compared with a published ES signature (Kauer data set).^28^ A more optimal gene expression profile for EF^Prx1^MSCL+Mcl1 sarcomas was prominent, when comparing relative expression levels of these signature genes in wtMSCL, EF^Prx1^MSCL, EF^Prx1^MSCL+Bcl2, EF^Prx1^MSCL+Mcl1 (Figures 5d and e) or EF^Prx1^MSCL+Bcl-x_*L*_ (data not shown) to human data. This suggests that transformation with MCL1 renders EF^Prx1^MSCL more similar to ES. We next examined whether on a transcriptomic level ES correlates better with the EF^Prx1^MSCL+Mcl1 transplant model than other human sarcomas using a comprehensive set of microarray data for different human sarcomas.^29^ From this data set normalized gene expression for each sarcoma was correlated with the log2 fold change of EF^Prx1^MSCL+Mcl1 *versus* wtMSCL. Although overall correlations to other sarcomas were low, the highest positive correlation (red bars) was seen for ES. This result suggests that among the tested sarcomas gene expression changes in the EF^Prx1^MSCL+Mcl1 as compared with wtMSCL is overall most similar to ES (Figure 5e). To determine functional categories of gene regulation we performed gene set enrichment analysis. Most prominently, we found different gene sets relating to cell cycle to be enriched in genes upregulated in the comparison EF^Prx1^MSCL+Mcl1 *versus* wtMSCL cells (Figure 5f), whereas the p53 signaling pathway was downregulated.

Tunnel and PI staining showed less tunnel-positive cells and more proliferation rate in EF^Prx1^MSCL+Mcl1 cell population, indicating the crucial role of Mcl1 for bypassing apoptosis in EF-expressing cells (Figure 5g; Supplementary Figure 7d). We noted similar amounts of immunostainig for key markers such as CC-3, Ki67, *β*-CATENIN, CYCLIN D1, CDK4/6 expression (Supplementary Figure 7g) in the compared groups upon quantification of the IHC as shown in Figure 5h. Western blot analysis displayed in average among 8 EF^Prx1^MSCL+Mcl1 tumors compared with two EF^Prx1^MSCL+Mcl1 or two EF^Prx1^MSCL expressing cells similar protein levels of CC-3 and reduced INK4A or P53 levels as quantified by densitometry (Supplementary Figure 7h). RB expression was lower, but pS780-RB expression was higher and CDK6 expression was also higher. Furthermore, sarcoma cells isolated from EF^Prx1^MSCL+Mcl1 tumors and recultivated displayed changed expression, most notable for upregulated p53, MCL1 and CDK6 expression. Interestingly, we observed a severe reduction of P19^ARF^ and P53 expression in the majority of eight analyzed tumors of the EF^Prx1^MSCL+Mcl1 group, whereas P19^ARF^ expression was lower in six tumors. In line, we also found a significant reduction of P16^Ink4A^ in both EF^Prx1^MSCL+Mcl1 cell lines and in the majority of EF^Prx1^MSCL+Mcl1 tumors. P19^ARF^ and P16^Ink4A^ were expressed lower in EF^Prx1^MSCL+Mcl1 tumor-derived cells and P53 expression was significantly enhanced in EF^Prx1^MSCL or even expressed/activated higher upon MCL1 transduction before transplant (Figure 5h). Total RB expression levels were slightly reduced (Supplementary Figure 7e).

### Blocked survival and proliferation arrests ES cell growth and induces apoptosis

CDK4 activity is required for cell cycle progression and it was shown that Mcl1 knockdown prolonged early G1 phase associated with decreased CDK4 expression.^30, 31^ Upon siRNA-mediated knockdown of *Mcl1* or *Cdk4* in Ewing-like mouse as well as in ES cell lines TC252 and SK-N-MC we could demonstrate that both genes are important for ES cell growth and survival (Figure 6). Mechanistically, we observed a slightly lower expression of pS780-RB after downregulation of *Mcl1* or *Cdk4*, whereas total RB levels were increased, indicating that *Mcl1* and *Cdk4* downregulation resulted in blocked proliferation (Figure 6a,Supplementary Figure 7i). Tumorigenic potential of siRNA-treated cells was assessed by colony-forming assay. The amount of *Mcl1* or *Cdk4* correlated with the number of colonies, indicating that MCL1 and CDK4 are required for efficient transformation. A siRNA-positive control targeting EF in EF^Prx1^MSCL+Mcl1 cells confirmed proliferation was EF-dependent (Figures 6a and b). Cell cycle analysis revealed that less *Mcl1* or *Cdk4* led to a prolonged G0/G1 and shortened S and G2/M phases (Figure 6c). To evaluate results of siRNA-mediated downregulation of *Cdk4* and to translate findings to pharmacologic targeting, we treated EF-dependent cells with Palbociclib, an FDA approved dual CDK4/6 inhibitor. Palbociclib (IC_50_=~1 *μ*M in human ES cell lines and IC_50_=~2 *μ*M in mouse EF-dependent cell lines) exposure led to reduced pS780-RB and increased total RB, whereas MCL1 levels were slightly decreased. Only a combination of CDK4/6 with the pan BCL2 family inhibitor Obatoclax resulted in significant growth inhibition of ES cells, whereas a BCL2 family inhibitor unable to target MCL1 (ABT-737) was inefficient to block proliferation (Figures 6d and e; Supplementary Figure 7j). Western blot analysis of treated human cell lines with Obatoclax and ABT-737 showed higher CC-3 intensity in cells treated with Obatoclax. The ES cell line T252 showed higher expression of CC-3 after treatment with ABT-737 (Supplementary Figure 8b).

## Discussion

Childhood cancer studies are greatly hampered by small study cohorts^32^ and an animal model to study ES is needed for preclinical drug testing and mechanistic insights into disease processes. We aimed to better model the cellular origin of ES through the use of *Prx1Cre*-driven EF expression. Moreover, we developed new primary cell models to study EF expression consequences on core cancer pathways such as apoptosis and cell cycle progression or bone developmental signaling pathways.^25, 26, 27, 33, 34, 35^ We conclude that EF expression blocks mesenchymal differentiation and it induces apoptosis. This cell death in the developing mesenchyme caused severe malformations in bone development with death in newborn owing to severe bone differentiation abnormalities, making a transplant model necessary. Therefore, we established a new *in vivo* transplant system to serve for drug testing studies and for mechanistic insights into key pathways driving sarcomagenesis.

ES cases in babies were reported^15, 16^ and therefore, our transgenic EF expression during limb differentiation could illuminate sarcoma formation in patients. We established multiple primary cell lines that were transformed to form sarcomas *in vivo* upon enforced BCL2 family member expression. We illuminated sarcoma formation through analysis and quantitation of key proteins involved in cancer progression. We found that our genetically engineered mouse model resembled sarcomas with close ES gene expression profile^28^ as determined by RNA-seq analysis, which could be useful to search for therapeutic intervention strategies. We found upregulated MCL1, CYCLIN D1, CDK4, but downregulated INK4A or P53 protein levels as prerequisites for ES proliferation and survival in line with similar findings in ES patients.^36, 37^

We observed an anterior-to-posterior differentiation defect, which could follow the wave of MSC dissemination in mammals that originate from neural crest. We noted deregulated WNT; HEDGEHOG, BMP and TGF-*β* pathways^17, 18, 19, 20, 21^ that culminated into skeletal development defects. Polydactyly was associated with elevated hedgehog signaling and *Gli1* expression known to be EF-dependent.^38^ Analysis of chondrogenesis and osteogenesis markers revealed an arrest of endochondral bone development. Inhibition of *Runx2*, *TgfbrI* or *TgfbrII* could be due to reported repression by EF.^39, 40^ Consequently, mature osteoblast markers lacked and TGF-*β*/BMP signaling was diminished. Normally, cartilage-derived *β*-catenin signaling promotes chondrocyte maturation and it is involved in ossification. BMP and TGF-*β* signaling are required for osteoblast and chondrocyte differentiation,^17, 20, 21, 41^ but bone invasion and osteolysis in ES are also associated with enhanced *β*-catenin signaling.^42, 43^ We observed downregulated BMP, TGF-*β* and *β*-catenin signaling at late development in EF^Prx1^ embryos, but high *β*-CATENIN expression was seen when sarcomas formed.

EF^Prx1^MSCL remained diploid despite high passages, but transformation did not occur. Interestingly, EF^Prx1^MSCL were immortal, but wtMSCL underwent senescence at low passage. Furthermore, despite contradictory literature, EF^Prx1^MSCL failed to differentiate, whereas wtMSCL differentiated normal.^5, 6, 7, 8^ EF-induced apoptosis was prominent in line with literature that identified *Procaspase 3* to be a direct target gene of EF.^11^ Higher expression of CASPASE-3 could be seen in liver and spleen of transgenic mice expressing EF.^10^ Introduction of EF in human mesenchymal progenitor can also induce prominently apoptosis.^44^

Enforced BCL2 family member expression was efficient to promote sarcomagenesis of transplanted EF^Prx1^MSCL. MCL1 resulted in highest similarity of tumor gene expression to human ES. Although survival is a core cancer pathway, the high protein expression of BCL2 family members in ES was so far neglected. Currently, we cannot rule out that a possible post-translation mechanism for high BCL2 family member protein expression could be responsible during Ewing sarcomagenesis. We conclude that overcoming high CASPASE-3-induced apoptosis will be important for transformation. Similarly, cell cycle deregulation in ES is also a consequence of transformation. A direct correlation between EF expression and the amount of cyclin D1 expression was shown^33, 34, 45^ and c-myc upregulation correlates with the Ki67 proliferation marker expression.^46^ We observed low expression of INK4A and/or P53 proteins in the majority of transplanted tumors from the MCL1 or BCL2 expressing cohort. Collectively, these results indicate a significant ES selection pressure for escape of apoptosis. Low expression of CDKN2A and/or P53 correlates with decreased apoptosis, or in case of CDKN2A loss also with enhanced self-renewal capacity of MSC.^36^ INK4A proteins are frequently lost owing to homozygous deletion or p53 mutations, both prominent in patients with ES.^37, 47^ Enhanced survival in collaboration with decreased pS780-RB expression and increased CDK4 levels could also boost transformation. It was shown that MCL1 and cell cycle progression are interconnected and more MCL1 expression accelerated the cancer cell cycle progression.^30, 31^ Here, we found that MCL1 knockdown led to a G1 cell cycle arrest by decreasing CYCLIN D1, CDK4/6 and by increasing P27 expression.^30, 31^ Enforced survival led to increased CDK4 expression and pRB phosphorylation. Knockdown of *Cdk4* or *Mcl1* in a panel of EF-dependent cell lines led to inhibition of cell proliferation and reduced colony formation. Targeting BCL2 family members displayed higher efficacy with Obatoclax *versus* ABT-737 treatment, but combination of Obatoclax with Palbociclib was most effective. Our findings extend and confirm also recent results that describe the requirement of ES cells for CYCLIN D1-CDK4/6 function.^35^

In summary, our findings propose that enhanced survival and proliferation with blocked mesenchymal differentiation are three prerequisites for Ewing Sarcoma formation. Our study displays mechanistic insights how the high apoptosis induced through EF-induced *Caspase-3* mRNA and protein expression can be overcome to promote sarcomas. We could show that pharmacologic inhibitors of CDK4/6 and BCL2 family members are more effective when combined as targeted inhibitors. Thus, new targeting approaches could be tried to counteract this metastasizing disease in a more efficient way.

## Materials and Methods

### Animal models and ethical approval

Transgenic *Rosa26-*EF^10^ were crossed to *Prx1Cre* mice.^13^ To isolate embryos vaginal plug checks were made, mice were separated and noon was counted as E0.5. Mice were kept under SBF conditions and animal experiments were approved (license number: BMWF-66009/0281-I/3b/2012). Immunocompromised NOD.Cg-PrkdcscidIl2rgtm1Wjl/SzJ (NSG) recipients were purchased (Harlan, United Kingdom).

### Cell culture, gene knockdown assay and inhibitor treatment

Cells were cultivated for inhibitor Palbociclib (PD-0332991) HCl in a dose–response cellular viability assay, incubated for 24 h (Selleckchem, Houston, TX, USA) with doses: 0, 0.3, 0.5, 1, 2, 5 and 7 *μ*M followed by viability counting using trypan blue. For inhibitor treatment viability values, IC_50_ was determined for human at 1 and for murine tumor cell lines up to 2 *μ*M. Treated cells were harvested for Western blot after 24 h treatment. For time-course assays, cells were seeded in tissue culture with inhibitors or vehicle (DMSO) up to 3 or 4 days. Ontarget Plus pool siRNAs for each individual gene were purchased and transfected as instructed (GE Dharmacon, Lafayette, CO, USA).

### *In situ* hybridization

Digoxigenin-labeled cRNA probes were generated by *in vitro* transcription of 1 *μ*g template DNA with RNA DIG labeling kit (Roche Diagnostics GmbH, Mannheim, Germany) according to manufacturer. *In situ* hybridizations were performed on serial paraffin sections as described.^48^ For each probe and time point, embryo sections were located for staining on one slide to allow for comparison.

### Quantitative immunostaining

Four precent formalin-fixed embryos were embedded in paraffin. Sections were processed prior to staining with specific antibodies (see Supplementary Table S2). Quantification of stained embryos was performed with one-way Anova test^23^ with Histo Quest analysis software (Tissue Gnostics GmbH, Vienna, Austria).

### Bioinformatic analysis

Illumina kits for strand-specific library preparation was used for RNA-seq and RNA was quantified using Qubit 2.0 Fluorometric Quantitation system (Life Technologies, Waltham, MA, USA). For comparison with human expression data orthologs were mapped using the biomaRt package (PMID:19617889). Gene set enrichment analysis was performed with java command line program (gsea2-2.0.13.jar) using the ‘preranked' method from the BROAD institute (PMID:16199517) and gene sets from MSigDb (http://software.broadinstitute.org/gsea/msigdb). Heatmap in Figure 5d: Mouse orthologs for genes in gene signature from^28^ were selected. Row-wise scaled, mean normalized expression levels for the four sample groups are shown. Genes in the heatmap are ordered by expression difference (ES tumor *versus* MSC) of human orthologs. Blue color indicates genes with lower expression in ES than in MSC, whereas red shows genes with higher expression in ES than in MSC. Correlation analysis: Sarcoma data from ref. 29 were filtered by excluding probe sets that had missing values in more than samples. Then for each gene the most variable probe set was selected and averaged per sarcoma entity.

### Statistical analysis

All results are presented as means±S.E.M. Data were considered statistically significant as described in each panel. All analyses were performed using Graph Pad Prism software (Graph Pad Software, La Jolla, CA, USA).

Further description for Bioinformatic analysis, tissue culture procedures, IHC and skeletal staining, FACS, qRT-PCR, primer table, specific antibody usage, transplant protocol and western blotting details please see Supplementary Data.

## Figures and Tables

**Figure 1:** EF expression blocks bone differentiation causing skeletal defects in EF^Prx1^ mice. (**a**) Scheme of the ROSA26-lox-STOP-lox-HA-hEWS/FLI1 transgenic mouse. (**b**) Representative picture of wt and EF^Prx1^ E16.5 embryo displays malformed limbs as indicated by black dashed circle. Skeletal preparations and analysis with Alcian Blue/Alizarin Red staining of E16.5 wt and EF^Prx1^. sc, scapula; hu, humerus; ra, radius; ul, ulna; ti, tibia; fi, fibula; fe, femur. (**c**) The list summarizes number of embryos (total, wt, EF^Prx1^) at different gestation days, and cumulative percentages/normal Mendelian ratio with indicated embryo numbers. (**d**) Histology analysis of E13.5 limbs stained by H&E or Van Kossa/Alcian Blue, which stains cartilage in blue and bone elements in red, indicated that there was no significant hypertrophic region present in EF^Prx1^ embryos in contrast to wt limbs. *RNA in situ* hybridization of E13.5 limbs confirmed an arrest in chondrocyte and osteoblast differentiation. For all embryos consecutive sections were performed. At least three different independent embryos for every single staining and for each time point were analyzed. Black circles indicate the magnified region showing in the lower row. (**e**) Detection of EF expression at the protein level at E16.5 using HA-tag antibody displayed significant transgenic protein product in limbs from EF mice. HSC-70 was used as a loading control. Fibro GFP or CRE: fibroblasts isolated from EF mice lentiviral-transduced with a construct containing GFP or the CRE recombinase was used as controls. Numbers of analyzed embryo/mice are indicated to corresponding images

**Figure 2:** Blocked bone signaling pathways upon EF expression. (**a** and **b**) Dimethylmethylene blue (DMMB) as a chondrocyte marker showed marked reduction of Glycosaminoglycan in mutant embryos. IHC staining analysis on consecutive embryo sections of E14.5 and postnatal day P1 mice showed that EF expression in limb mesenchyme promotes downregulation of TGF-*β* signaling pathway. Black circles indicating the magnified region showing in the next column. (**b**) Quantification of IHC signals from (**a**). At least three different independent embryos for every single staining and for each time point were carried out. Quantitation was done by (ANOVA) one-way analysis of variance. *P<0.5, **P<0.05 and ***P<0.005

**Figure 3:** EF expression induces apoptosis and leads to diminished cell cycle progression. (**a**) HA-tag staining was performed to detect the EF translocation product. The rate of proliferation was comparable to wt based on Ki67 proliferation marker staining. TUNEL staining displayed highly elevated apoptosis at P1. (**b**) P21 (CDKN1A) protein level was upregulated. Prominent nuclear staining of P21 at E14.5, decreased at E16.5 and P1. cyclin D1 expression was decreased during development till P1. Black circles indicating the magnified region showing in the next column. (**c**) Quantification of IHC from part A and B. At least three different independent embryos of wt or mutant for every single staining and for each time point were analyzed. Experimental staining results were evaluated using (ANOVA) one-way analysis of variance. Insets in separate panel highlight cellular details. *P<0.5, **P<0.05 and ***P<0.005

**Figure 4:** EF^Prx1^ mesenchymal stem cells like cells (EF^Prx1^MSCL) are immortal, but display high apoptosis and fail to differentiate. (**a**) MSCL were isolated from P1 mouse long bone cartilaginous elements of wt or EF^Prx1^ newborns (left). A representative primary cell line from low passage 3–4 in case of wtMSCL or passage 8–10 in case of EF^Prx1^MSCL line is shown. WtMSCL were able to differentiate along mesenchymal lineages, whereas EF^Prx1^MSCL failed to differentiate. Differentiation was induced as detailed in Materials and Methods to obtain osteocytes (stained with Alizarin red), chondrocytes (Van Kossa staining) and adipocytes (Oil red O staining). An example from three independent differentiation experiments is shown (right). (**b**) Western blot analysis (*n*=2, each) of HA-tag and qRT-PCR (*n*=6, each) proved significant EF transgene expression. The EF^Prx1^MSCL displayed high surface expression of CD90 (Thy-1.1; *n*=3, each), a MSC marker, compared with wtMSCL. (**c**) EF^Prx1^MSCL has blunted TGF-*β* signaling as measured by reduced expression levels of *TgfbrI, TgfbrII* and *Dlx5.* Similarly, osteogenic markers like *Osx*, *Sox9* and *Osc* were expressed to lower levels, but enhanced hedgehog signaling was found as evident by higher *Ihh*, *Smo* and *Gli1* expression using qRT-PCR. Error bars represent S.E.M. of six individual measurements. All qRT-PCR results were normalized to *Gapdh*. For wt or mutant embryos at least three different independent experiments were carried out. (**d**) Representative cell cycle analysis of six wtMSCL (passage 3) or 12 EF^Prx1^MSCL at early (passage 8) or late (passage 55) culture time as measured by propidium iodide (PI) staining. *Caspase-3* expression was induced in EF^Prx1^MSCL as measured by qRT-PCR compared with wtMSCL levels causing high apoptosis. *P<0.5, **P<0.05 and ***P<0.005

**Figure 5:** EF^Prx1^MSCL give rise to sarcomas upon enhanced expression of anti-apoptotic BCL2 family members. (**a**) ES cell lines SK-N-MC, TC71, TC252 and A673 expressed prominent level of MCL1, BCL2 and BCL-x_*L*_. Colorectal carcinoma cell lines HT29, HCT116, SW620 and LS174T were used as positive control. CDK4 expression was higher than in the control human prostate epithelial cell line RWPE-1. (**b**) Four different EF^Prx1^MSCL and four different wtMSCL were transduced by retrovirus with either GFP-vector, Bcl2-IRES-eGFP, Bcl-x_*L*_-IRES-eGFP or Mcl1-IRES-eGFP. A total of 12 primary cell transductions for each cell line were xenografted (*n*=12, each). All Bcl2, Bcl-x_*L*_ and Mcl1-expressing EF^Prx1^MSCL lines formed reproducibly sarcomas with full penetration as quantified in the right graph. None of the controls like the wtMSCL with or without BCL2 family member transduction or GFP-transduced EF^Prx1^MSCL formed any sarcoma up to 6 months post transplant. (**c**) Xenografted sarcomas were positive for periodic acid schiff (PAS) and neuronal-specific enolase (NSE) staining. SK-N-MC xenograft served as positive control. (**d**) RNA-seq analysis (from left to right) of wtMSCL, EF^Prx1^MSCL, two sarcoma samples from EF^Prx1^MSCL+Bcl2 and EF^Prx1^MSCL+Mcl1 revealed that samples become more similar to the ES gene expression signature (Kauer data set^28^). (**e**) Clustering analysis showed the best matching of EF^Prx1^MSCL+Mcl1 tumor genes to human ES signatures. (**f**) Gene enrichment analysis (GSEA) exhibited a noticeable upregulation of cell cycle and a downregulation of p53 pathway in mouse EF^Prx1^MSCL+Mcl1 tumors *versus* wtMSCL. (**g**) EF^Prx1^MSCL at passage 30 served as controls. Two representative sarcoma lines EF^Prx1^MSCL+Mcl1 were established each that displayed an increase of GFP expression and a decrease in TUNEL^+^ cells after sarcomas formed, whereas PI staining displayed more proliferation in EF^Prx1^MSCL+Mcl1 and EF^Prx1^MSCL+Mcl1 tumor-derived cells. (**h**) Proliferative sarcoma cells were also positive for nuclear *β*-catenin, cyclin D1, CDK6 and CDK4, whereas cleaved caspase-3 (CC-3) was downregulated. All shown staining images are a representative of independent IHC analyses of *n*=12 isolated tumors per group. (**i**) Western blot of two EF^Prx1^MSCL, two EF^Prx1^MSCL+Mcl1, eight EF^Prx1^MSCL+Mcl1 sarcomas and two EF^Prx1^MSCL+Mcl1 tumor-derived cells showed an overall reduced level of caspase-3 (Pro CC-3), CC-3, P16^Ink4A^, P19^ARF^, P53 and higher amount of pS780-RB protein level upon enforced MCL1 expression in EF^Prx1^MSCL and associated tumor samples. Representative blots of three independent analyses are shown

**Figure 6:** Knockdown of Mcl1 or Cdk4 induced cell cycle arrest and inhibited ES cell proliferation. (**a**) Mcl1 and Cdk4 siRNA analysis and expression check in murine and human ES cell lines resulted in upregulation of total RB and lower amount of pS780-RB. (**b**) Colony-forming assay in matrigel displayed reduced clonogenic potency of EF-dependent cell lines after knockdown of Mcl1 or Cdk4 by siRNA treatment. (**c**) Cell cycle analysis of Mcl1 or Cdk4 siRNA treatment displayed enhanced G1 arrest. (**d**) *In vitro* growth inhibition of mouse and human EF-dependent cell lines by Palbociclib as well as the combinatorial treatment of Palbociclib and Obatoclax in triplicate. Cells were treated with inhibitors at the indicated concentration for 24 h. (**e**) CDK4/6 inhibition by Palbociclib displayed similar results as seen in the CDK4 siRNA assay

## Abbreviations

BCL2: B-cell lymphoma 2
BCL-x_*L*_: BCL2-like 1 isoform 1
BMP: bone morphogenetic protein
CC-3: cleaved caspase-3
CDK4: cyclin-dependent kinase 4
CDK6: cyclin-dependent kinase 6
CDKN1A: cyclin-dependent kinase inhibitor 1A
Col2a1: collagen 2a1
Col10a1: collagen 10a1
Col1a1: collagen 1a1
DLX5: distal-less homeobox 5
DMMB: dimethylmethylene blue
ES: Ewing sarcoma
EF: EWS/FLI1
ERG: V-Ets avian erythroblastosis virus E26 oncogene homolog
EWS: Ewing Sarcoma breakpoint region
FDA: Food and drug administration of USA
FLI1: friend leukemia virus integration 1
GAPDH: glyceraldehyde-3-phosphate dehydrogenase
HSC-70: heat shock protein 70
Ihh: Indian hedgehog
INK4A (CDKN2A): cyclin-dependent Kinase 4 Inhibitor A
IRES: internal ribosome entry site
Mcl1: myeloid cell leukemia 1
MSC: mesenchymal stem cell
NSE: neuronal-specific enolase
Osxo: osterix
Osc: osteocalcin
PAS: periodic acid Schiff
PI staining: propidium iodide
pRB: protein Retinoblastoma 1
Prx1: paired related homeobox 1
Runx2: runt-related transcription factor 2
SMAD1/4/5/7: mothers against decapentaplegic homolog 1/4/5 or 7
Smo: smoothened
Sox9: sex determining region Y-box 9
TGF-*β*: transforming growth factor beta
TGF-*β*r1/2: transforming growth factor beta receptor 1 or 2
TUNEL: terminal deoxynucleotidyl transferase dUTP nick end labeling
Wt: wild type
WNT: wingless-type MMTV integration site family member
